# Study on the Effect of Straw Mulching on Farmland Soil Water

**DOI:** 10.1155/2022/3101880

**Published:** 2022-09-29

**Authors:** Jin-Xia Zhang

**Affiliations:** College of Water Conservancy and Hydropower Engineering, Gansu Agricultural University, Lanzhou, 730070 Gansu, China

## Abstract

Straw mulching farming is currently an effective dry farming technique for improving arid soil environments. Straw mulching technology can increase the infiltration capacity of soil water and improve crop yield and water use efficiency. In this study, the aim is to improve the soil water holding capacity, water retaining capacity, and comprehensive water use efficiency of crops in dry farmland. First, the response surface model is used to study and analyse the optimal parameters of straw returning and its mulching technology, and then, the crop yield, water consumption, and comprehensive water use efficiency of spring corn under different mulching conditions during 2017-2019 are studied. The test results show that the optimized parameters obtained by the response surface model are as follows: film thickness is 0.03 mm, straw returning amount is 4500 kg/hm^2^, straw particle size is 5 mm, and straw returning depth is 25 mm. At this time, the maximum soil water storage can reach 404.50 mm. The results of the straw mulching test show that under 4500 kg/hm^2^ mulching, the soil has more water storage, higher soil water content, and a simultaneous increase in water consumption, which is conducive to the efficient use of limited precipitation by crops. The field experiment for three years shows that 4500 kg/hm^2^ straw (wheat) mulching in the dry farming area of southern Ningxia can better store water and protect soil moisture, promote the virtuous cycle of farmland soil water, and show outstanding performance in improving corn yield and water use efficiency, which can be popularized and implemented in spring corn production in this area.

## 1. Introduction

Straw return to the field is an effective field fertilization technology to improve soil moisture, physical and chemical properties, and fertility to improve crop yield and quality. Straw return to field technology can not only solve the environmental pollution and resource waste caused by straw burning and stacking but also greatly promote the sustainable, circular, and healthy development of the rural planting industry [1–4]. Straw mulching farming is currently an effective dry farming technique for improving arid soil environments. Straw mulching technology can strengthen the accumulation of soil organic matter, increase soil water infiltration capacity and effective reservoir capacity, adjust soil temperature, improve crop yield and water use efficiency, etc. [5, 6]. However, the effects of straw mulching techniques on crop yields are quite different under different amounts of straw mulch, different soil types, and different tillage practices, and yield reductions under crop protection tillage practices have distinct regional characteristics [7]. In addition, some studies show that an unreasonable mulching amount and method can easily produce negative effects on crop growth and development, which leads to yield reduction. Therefore, the main problems existing in straw returning and mulching technology need to be further studied [8–10].

Based on this, this study selects the dry farming area in southern Ningxia as the research area, aimed at improving the soil water holding capacity and retaining capacity and comprehensive water use efficiency of crops. First, the response surface model is used to study and analyse the optimal parameters of straw returning and its mulching technology. Based on the optimal parameters, spring corn crops are selected as the research object, and the crop yield, water consumption, and comprehensive water use efficiency of spring corn under different mulching conditions during 2017-2019 are studied to provide a theoretical basis for the promotion and application of straw mulching technology in this type of region.

## 2. Materials and Methods

### 2.1. Overview of the Test Area

In this study, the dry farming area in southern Ningxia is selected as the research area. The annual precipitation in the selected test area is approximately 400-500 mm, and the rainy season is concentrated in the four months of June, July, August, and September. The selected area is rich in light and heat resources, with an average annual temperature of 6-15°C. The selected soil is loess. The average bulk density of the soil at a depth of 0-50 cm is 1.25 g/cm^3^, the pH value of the soil varies from 7.6 to 8.1, the field water holding capacity is approximately 25.33%, the fertility is relatively low, and the contents of organic matter and total nitrogen in the soil are approximately 8.03 g/kg and 0.36 g/kg, respectively. The selected research time was three consecutive years from 2017 to 2019, and the effective rainfall of crops in the sowing and seedling periods was 270.9 mm, 294.2 mm, and 366.5 mm, respectively.

### 2.2. Test Scheme Design

In this study, spring corn was selected as the test variety, and the field planting test was carried out by film mulching+straw mulching. Before the formal test, the interaction rule between the parameters, such as film thickness, straw returning amount, straw particle size, and straw returning depth, used in straw returning to the field was analysed by the response surface model to obtain the optimal parameters of straw returning to field (the design of test parameters is shown in Table 1).

Then, using the optimized parameters, a test on soil water consumption and crop water comprehensive use efficiency with different straw mulching amounts was carried out. The test took planting without straw mulching as a control (CK), and then, with other parameters unchanged, the straw mulching amounts of 3000 kg/hm^2^ (E1), 4500 kg/hm^2^ (E2), and 6000 kg/hm^2^ (E3) were taken as test groups, and each group was repeated three times at random.

### 2.3. Test Items and Data Statistics

The main indexes tested in this study mainly include soil water storage, crop water consumption, and the comprehensive water use efficiency of crops [11–13], and the calculation formulas of each index are as follows:

1. Soil water storage is an important index reflecting the water storage capacity of soil, and its calculation formula is

(1) $$\begin{array}{c} W=\frac{\left(H\times A\times B\times 10\right)}{100}. \end{array}$$

*W* is the soil water storage, mm; *H* is the soil depth, cm; *A* is the soil bulk density, g/cm^3^; and *B* is the soil water content, %.

(2) Crop water consumption (ETa) reflects the water consumption of crops in the growth process, and its calculation formula is

(2) $$\begin{array}{c} \text{ETa}=\text{SG}+P+W_{1}-W_{2}-R-D. \end{array}$$

ETa is crop water consumption, mm; SG is groundwater consumption, mm; *W*_1_ is soil water storage before sowing, mm; *W*_2_ is soil water storage after harvest, mm; and *R* and *D* are runoff and leakage, respectively, mm.

(3) WUE is a vital index reflecting the relationship between crop material production and water consumption. The calculation formula is

(3) $$\begin{array}{c} \text{WUE}=\frac{Y}{ETa}. \end{array}$$

WUE is the comprehensive use efficiency of crops, kg/(mm·hm^2^); *Y* is crop yield, kg/hm^2^; and ETa is soil water consumption.

## 3. Results and Analysis

### 3.1. Optimization of the Straw Mulching Scheme in Farmland Soil

#### 3.1.1. Mathematical Modelling

Taking film thickness *A*, straw returning amount *B*, straw particle size *C*, and straw returning depth *D* as four influencing factors of the response surface model and taking the soil water storage amount before sowing *R* as the response value, Design-Expert 10 software was used to design a four-factor three-level test to discuss the interaction rules of each process parameter on soil water storage under straw mulching. The test design results are shown in Table 2. It can be seen from the table that within the selected parameter range, the change range of soil water storage is 303.5 mm~395.6 mm.

#### 3.1.2. Variance Result Analysis

According to the Box-Behnken Design (BBD) in the response surface method, variance analysis of the test model was carried out, and the results are shown in Table 3. It can be seen from the data in the table that the binary multiple regression model of soil water storage has *F* = 28.77, *P* < 0.01, which indicates that the model has significant differences and can be used to optimize the test parameters of soil water storage under straw mulching. In this study, the best response surface model was obtained by regression analysis of the above data, using soil water storage *R* as the objective function. Then, the insignificant items in the model were eliminated to obtain the final model, and its quadratic multiple regression equation was *R* = 358.08 + 33.57*A* + 12.92*B* − 3*C* + 4.52*D* − 4.8*AB* + 9.17*CD*.

#### 3.1.3. Result Analysis of the Response Surface Model

*(1) Interaction of Film Thickness and Straw Returning Amount on Soil Water Storage*.  Figure 1 is the response surface model of film thickness and straw returning amount to the soil water storage under straw mulching. It can be seen from the figure that under the condition of keeping straw particle size and straw returning depth unchanged, the soil water storage gradually increases with the increase in film thickness while showing a trend of first rising sharply and then increasing gently with the increase in straw returning amount. The use of mulching can reduce the evaporation rate of water to a certain extent, and the mulching rate gradually decreases with increasing film thickness so that the soil water retaining capacity increases, and the water storage also increases [14]. On the other hand, with the same film thickness, the increase in straw returning amount can significantly improve the soil water holding capacity, which makes the soil water storage increase with the increase in straw returning amount, but when it increases to a certain extent, the soil water storage will not further increase [15]. In addition, from the contour map, it can be clearly observed that the effect of the amount of returned straw on soil water storage is significantly higher than that of film thickness, and the interaction between them is obvious.

*(2) Interaction of Film Thickness and Straw Particle Size on Soil Water Storage*.  Figure 2 shows the response surface model of film thickness and straw particle size to soil water storage. It can be seen from the figure that with the same straw returning amount and straw returning depth, the soil water storage increases slowly with increasing film thickness, while it shows a trend of first increasing and then slowly decreasing with increasing straw particle size. To some extent, the increase in straw in the soil will affect the contact area between the soil particles and change the bulk density of the soil. In this test, with the increase in straw particle size, the compactness of the soil will decrease, and the pore structure will increase, so the bulk density will also decrease, resulting in an increase in the soil water holding capacity. Then, the straw particle size continues to increase, but the soil water holding capacity decreases to a small extent because although the bulk density of the soil is reduced with larger particle size, the dissipation space of water molecules in the soil also increases, and the soil water retaining capacity decreases, so the soil water holding capacity decreases [16, 17]. In addition, from the contour map, it can be found that the effect of film thickness and straw particle size on soil water storage is basically the same, and the interaction between them is not obvious.

*(3) Interaction of Straw Returning Amount and Straw Particle Size on Soil Water Storage*.  Figure 3 shows the response surface model of the straw returning amount and straw particle size to soil water storage. It can be seen from the graph that, keeping film thickness and straw return depth constant, soil water storage increases sharply and then slows down as the amount of straw returned to the field increases, while an increase in straw particle size causes soil water storage to increase and then decrease. Combined with the contour map and 3D model, it can be seen that the difference in the effect of the amount of returned straw on the soil water storage is more obvious than that of the straw particle size. In addition, there is an obvious interaction between the straw returning amount and straw particle size, which forms a “climbing” shape between them.

*(4) Interaction of Straw Particle Size and Straw Return Depth on Soil Water Storage*.  Figure 4 shows the response surface model of straw particle size and straw returning depth to soil water storage. It can be seen from the figure that under the condition of constant film thickness and straw returning amount, the soil water storage increases first and then decreases with the increase in straw particle size and decreases gently with the increase in straw returning depth. Due to the difference in water content at different soil depths, the straw returning depth will also affect the soil water storage to a certain extent. In this test, the soil water content slightly decreases with increasing soil depth, but the decrease difference is not obvious, which also makes the difference in soil water storage between the parameters of returning depth not obvious [18, 19]. In addition, it can be seen from the contour map that there is a certain degree of interaction between straw particle size and straw returning depth, but the interaction is not significant.

In summary, to improve the soil water storage, by response surface model analysis, the optimized process parameters obtained by this study are as follows: film thickness 0.03 mm, straw returning amount 4500 kg/hm^2^, straw particle size 5 mm, and straw returning depth 25 mm. At this time, the maximum soil water storage can reach 404.50 mm.

### 3.2. Effects of Different Straw Mulching Amounts on Water Consumption and Water Use Efficiency of Farmland Crops

#### 3.2.1. Trends in Crop Yield

The crop yield during the three years is shown in Table 4. It can be seen from the table that the effects of different straw mulching treatments on crop yield are obviously different in the three-year period. In 2017, the crop yields of the E1, E2, and E3 treatment groups increased by 2.94%, 13.79%, and 16.69%, respectively, compared with the CK group. In 2018, the crop yields of the E1, E2, and E3 treatment groups increased by 13.66%, 23.27%, and 29.03%, respectively, compared with the CK group. In 2019, the crop yields of the E1, E2, and E3 treatment groups increased by 6.81%, 12.46%, and 18.18%, respectively, compared with the CK group. After three years, the E2 and E3 treatment groups showed significant differences compared with the control group (*P* < 0.05), while E1 showed no significant difference compared with the control group (*P* > 0.05). It is worth noting that under the same test treatment, the precipitation in the growth period of crops in 2018 was higher than that in 2017, but the crop yield was lower, which may be due to the severe drought in the first quarter of 2018, affecting the growth of crops in the seedling period. Although there was more rain in the second quarter, it was not enough to completely compensate for the negative impact of the previous drought on crop growth [20].

#### 3.2.2. Trends in Soil Water Consumption

Under the influence of precipitation distribution and ambient temperature, the water consumption of crops in different years is also different (as shown in Table 4). The rainfall period in 2017 was mainly distributed in the early stage of crop growth, so the water consumption of crops under each test condition was E3 > E2 > CK > E1, among which the difference between the E1 and CK treatment groups was not obvious (*P* > 0.05), while compared with CK, the difference between E2 and E3 was obvious (*P* < 0.05). The rainfall period in 2018 was mainly distributed in the middle and late stages of crop growth, so the water consumption of crops under each test condition treatment was E3 > E2 > E1 > CK, and the water consumption of each test treatment increased by 30.3 mm, 29.6 mm, and 12.1 mm, respectively, among which the difference between the E2 and E3 treatment groups was obvious compared with the CK group (*P* < 0.05). In 2019, the rainfall period was evenly distributed, and the water consumption of crops under each test condition was E2 > E3 > E1 > CK. Compared with the CK group, the water consumption of each test treatment increased by 17.5 mm, 14.3 mm, and 9.7 mm, respectively, but there was no significant difference between the E2 and E3 treatment groups (*P* > 0.05).

#### 3.2.3. Trends in Comprehensive Water Use Efficiency of Crops

Comprehensive water use efficiency is an index used to evaluate the growth and decline relationship among crop yield, transpiration water consumption, and surface water evaporation. Table 4 shows that in 2017, the comprehensive water use efficiency of the E3, E2, and E1 test groups increased by 9.10%, 7.36%, and 4.98%, respectively, compared with that of the CK group. In 2018, the comprehensive water use efficiency of the E3, E2, and E1 test groups increased by 14.77%, 9.90%, and 8.26%, respectively, compared with that of the CK group. In the past two years, the differences between the E3 and E2 treatment groups were significant (*P* < 0.05), E1 was not significant (*P* > 0.05), and E3 and E2 and E1 had no significant differences between the CK group (*P* > 0.05). In 2019, the comprehensive water use efficiency of each treatment group increased by 11.84%, 7.52%, and 3.57% compared with CK, among which E3 and E2 had significant differences compared with CK (*P* < 0.05), while E1 had no significant differences (*P* > 0.05), and E3 and E2 and E1 had no significant differences between the CK groups (*P* > 0.05).

In summary, under 4500 kg/hm^2^ mulching, the soil has more water storage, higher water content, and higher water consumption, which is conducive to the efficient use of limited precipitation by crops, thus increasing the spring corn yield. Field experiments over three years show that 4500 kg/hm^2^ straw (wheat) mulching in the dry farming area of southern Ningxia can better store water and protect soil moisture, promote the virtuous cycle of farmland soil water, and show outstanding performance in improving corn yield and water use efficiency, which can be popularized and implemented in spring corn production in this area [21, 22].

## 4. Conclusion

- The test results show that the optimized parameters obtained by the response surface model are as follows: film thickness is 0.03 mm, straw returning amount is 4500 kg/hm^2^, straw particle size is 5 mm, and straw returning depth is 25 mm. At this time, the maximum soil water storage can reach 404.50 mm
- The field experiment for three years shows that 4500 kg/hm^2^ straw (wheat) mulching in the dry farming area of southern Ningxia can better store water and protect soil moisture, promote the virtuous cycle of farmland soil water, and show outstanding performance in improving corn yield and water use efficiency, which can be popularized and implemented in spring corn production in this area

## Figures and Tables

**Figure 1:** Contour map and 3D model of the effect of film thickness and straw returning amount on soil water storage.

**Figure 2:** Contour map and 3D model of the effect of film thickness and straw particle size on soil water storage.

**Figure 3:** Contour map and 3D model of the effect of straw returning amount and straw particle size on soil water storage.

**Figure 4:** Contour map and 3D model of the effect of straw particle size and straw returning depth on soil water storage.

**Table 1:** Factor level design scheme of the response surface method.

Experiment factor	Coded value	Factor level and coding design		
		-1	0	1
Film thickness (mm)	*A*	0.01	0.02	0.03
Straw returning amount (kg/hm^2^)	*B*	3000	4500	6000
Straw particle size (cm)	*C*	3	5	7
Straw returning depth (cm)	*D*	15	25	35

**Table 2:** Response surface test design and results.

Test number	Influencing factors				Soil water storage (*R*)
	Film thickness (*A*)	Straw returning amount (*B*)	Straw particle size (*C*)	Straw returning depth (*D*)	
1	0.01	4500	5	35	320.8
2	0.03	4500	7	25	395.6
3	0.03	4500	3	25	392.5
4	0.02	4500	5	25	357.6
5	0.02	4500	7	35	375.6
6	0.03	3000	5	25	383.5
7	0.02	4500	5	25	360.2
8	0.02	6000	5	15	370.3
9	0.03	4500	5	15	386.7
10	0.01	4500	5	15	325.4
11	0.02	3000	5	15	340.5
12	0.01	3000	5	25	303.5
13	0.02	3000	7	25	342.4
14	0.02	6000	5	35	374.2
15	0.02	4500	5	25	358.4
16	0.02	4500	5	25	356.7
17	0.02	3000	5	35	346.2
18	0.03	6000	5	25	390.5
19	0.02	4500	5	25	357.5
20	0.02	4500	3	35	370.8
21	0.01	6000	5	25	329.7
22	0.02	6000	7	25	373.2
23	0.03	4500	5	35	390.4
24	0.02	3000	3	25	345.6
25	0.01	4500	7	25	326.9
26	0.02	4500	7	15	334.5
27	0.01	4500	3	25	330.1
28	0.02	6000	3	25	378.8
29	0.02	4500	3	15	366.4

**Table 3:** Variance analysis results of soil water storage under straw mulching.

Source	Sum of squares	df	Mean square	*F* value	*P* value
Model	16593.83	14	1185.27	28.77	<0.0001^∗∗^
*A*—film thickness	13520.65	1	13520.65	328.17	<0.0001^∗∗^
*B*—straw returning amount	2002.08	1	2002.08	48.59	<0.0001^∗∗^
*C*—straw particle size	108	1	108	2.62	0.1277
*D*—straw returning depth	244.8	1	244.8	5.94	0.0287^∗^
*AB*	92.16	1	92.16	2.24	0.157
*AC*	9.92	1	9.92	0.24	0.6312
*AD*	17.22	1	17.22	0.42	0.5284
*BC*	1.44	1	1.44	0.035	0.8544
*BD*	0.81	1	0.81	0.02	0.8905
*CD*	336.72	1	336.72	8.17	0.0126
*A* ^2^	46.5	1	46.5	1.13	0.306
*B* ^2^	35.14	1	35.14	0.85	0.3714
*C* ^2^	126.87	1	126.87	3.08	0.1011
*D* ^2^	2.32	1	2.32	0.056	0.816
Residual	576.8	14	41.2		
Lack of fit	569.74	10	56.97	32.24	0.0022
Pure error	7.07	4	1.77		
Cor total	17170.63	28			

Note: ∗ indicates a significant difference, *P* < 0.05; ∗∗ indicates extremely significant.

**Table 4:** Crop yield, water consumption, and comprehensive water use efficiency under different test conditions in the last three years.

Year	Treatment	Yield (kg/hm^2^)	Water consumption (mm)	WUE (kg/(mm·hm^2^))
2017	CK	4768.65	276.3	17.26
	E1	4908.7	270.9	18.12
	E2	5426.43	292.8	18.53
	E3	5564.34	295.5	18.83

2018	CK	4307.65	243.8	17.67
	E1	4896.24	255.9	19.13
	E2	5309.85	273.4	19.42
	E3	5558.27	274.1	20.28

2019	CK	5699.78	308.2	18.49
	E1	6087.72	317.9	19.15
	E2	6409.88	325.7	19.88
	E3	6736.12	322.5	20.68

## Data Availability

The labeled dataset used to support the findings of this study are available from the corresponding author upon request.
